# Malaria Infection, Parasitemia, and Hemoglobin Levels in Febrile Patients Attending Sibu Sire Health Facilities, Western Ethiopia

**DOI:** 10.1155/2022/6161410

**Published:** 2022-08-12

**Authors:** Gobena Bayisa, Mebrate Dufera

**Affiliations:** Department of Biology, College of Natural and Computational Sciences, Wollega University, Nekemte, Ethiopia

## Abstract

**Background:**

Malaria is endemic in tropical and subtropical regions and causes up to one million deaths each year. It mostly affects sub-Saharan African countries including Ethiopia. In Ethiopia, it was estimated that about 75% of the land and 68% of the population are exposed to malaria. The aim of the current study was to determine malaria cases, its impact on the level of hemoglobin, and parasitemia and predisposing factors among febrile patients who visited Sibu Sire Health Care centers.

**Methods:**

Institution-based cross-sectional study was undertaken from May to October, 2020. Febrile patients who visited Sibu Sire Health Care centers were purposefully selected as the target population for the present study. Blood samples were collected and thick and thin smears stained with Giemsa. Hemoglobin level was determined using HemoCue Hb 301. Structured questionnaire and SPSS statistical software were used to collect and analyze data. *P* value < 0.05 was stated as statistically significant.

**Results:**

The overall prevalence of malaria was 168/979 (17.2%) out of which *Plasmodium falciparum* was 132/168 (78.5%), *Plasmodium vivax* was 27/168 (16.1%), and mixed infection was 9/168 (5.4%). To assess factors associated with dependent variable and determine the strength of association, binary logistic regression was used at adjusted odds ratios with 95% confidence intervals. The associations between malaria cases, hemoglobin levels, and parasitemia were estimated to evaluate the impacts of malaria on hemoglobin levels and parasitemia level. Out of 979 febrile patients (male 453 and female 526), 168 (male 99 and female 69) individuals were infected with *Plasmodium* species and *Plasmodium falciparum* were the predominant parasites. The majority of the study participants 144/168 (85.7%) were from rural residences. Highest malaria-infected patients 74/168 (44%) were aged between 15 and 30 years old. The level of hemoglobin and parasitemia was highly associated with malaria cases; hence, in this study area, intensities of hemoglobin and parasitemia are significantly associated with *Plasmodium* species.

**Conclusion:**

There was a moderate prevalence of malaria parasitemia and hemoglobin level among patients visiting Sibu Sire Health Care center; however, it needs further intervention to prevent and control malaria transmission in this malaria hotspot area.

## 1. Introduction

Malaria is a disease caused by protozoan parasites of *Plasmodium* species which are transmitted by infected female anopheles mosquito. Still malaria remains a major public health problem causing a significant morbidity and mortality. Globally, in 2018, an estimated of 228 million cases of malaria occurred with 405,000 deaths, and sub-Saharan Africa (SSA) accounted for 216 million cases and 445,000 deaths mostly in young children [1]. The vast majority of deaths are caused by *P. falciparum*, while *P. vivax*, *P. malariae*, and *P. ovale* cause generally milder forms of malaria [2].

Ethiopia is one of the most malaria endemic countries [3]. About 68% of the Ethiopian population resides in the area below 2000 m and considered to be at risk of malaria. Among the five types of *Plasmodium* parasites that cause malaria, *Plasmodium vivax* and *Plasmodium falciparum* are widely distributed in Ethiopia [1]. In the country, malaria transmission occurs with the highest transmission period from June to September [4]. Malaria transmission is highly seasonal throughout the country that depends on altitude and climatic variations [5].

Various retrospective cross-sectional studies conducted in parts of the Oromia region and western parts of Ethiopia have shown the overall malaria positivity rates ranging from 0.56% to 49.4%. Specifically, in the East Wollega Zone, Western Oromia, malaria has widespread occurrence and is a major public health burden [6].

A ten-year retrospective malaria trend analysis conducted in Sibu Sire by Gemechu et al. in Western Ethiopia [7] showed that among a total of 30,070 collected blood films, 20.07% of them become positive for malaria. The highest malaria case 31.2% was recorded in 2004 followed by 2010 and 2005 at a prevalence rate of 13.7% and 13%, respectively. Furthermore, with different fluctuation rates, the highest peak was in June at a prevalence rate of 18.9%, followed by May, November, and July with a prevalence of 13.3%, 13.2%, and 11.2%, respectively. Although the population of Sibu Sire is vulnerable to malaria, so far there is no published report of febrile patients regarding malaria cases and its impacts. Therefore, this study was aimed at assessing malaria cases, its impacts, and associated risk factors among febrile patients visiting Sire Primary Hospital and health centers.

## 2. Methods

### 2.1. Study Area

The study was conducted in Sibu Sire District, East Wollega Zone of Oromia Regional State, Western Ethiopia. The area is located 281 km west from Addis Ababa and 50 km east from Nekemte, the administration town of the East Wollega Zone. It has a total population of 172,573 [8], an altitude between 1300 and 3020 meters above sea level with a latitude of 9°04′60.00^″^N and longitude of 36°49′59.99^″^E, mean temperature of 22.55°C, and annual average rainfall of 1295 mm [9]. The existing health facilities rendering health services in the town include one Hospital, four health centers, seven middle-level clinics and 13 small private clinics, five drug stores and supplies, three pharmacies, and five rural drug venders. Of these, Sire and Chingi health centers as well as Sire Primary Hospital who serves both the urban and rural residents were selected as the study area of this research work which is attributed to the presence of laboratory facilities such as electricity, microscope, and HemoCue Hb 301.

### 2.2. Study Design and Period

Facility-based cross-sectional study was conducted involving febrile patients who visited the Sibu Sire health center, Chingi health center, and Sire Primary Hospital from May 2020 to October 2020. The study involved laboratory examination of blood film for detections of malaria parasites.

### 2.3. Study Population

All febrile patients 979 (male 453 and female 526) in Sibu Sire District who visited the Sibu Sire health center, Chingi health center, and Sire Primary Hospital were included in the study. Ethical clearance was obtained from the Wollega University Research Ethics Review Committee.

### 2.4. Inclusion and Exclusion Criteria

The inclusion criterion was any febrile patients visiting the Sibu Sire health center, Chingi health center, and Sire Primary Hospital for fever treatment and interested to join the study.

The exclusion criterion was febrile patients who are under malaria medication in the same week.

### 2.5. Sample Size Determination and Sampling Techniques

All available and eligible febrile patients who visited Sibu Sire Health care centers and hospital were included in the study. A nonprobability sampling technique was used to select febrile patients coming to the health center for blood film examination. An active case detection sample was collected.

## 3. Method of Data Collection

### 3.1. Blood Sample Collection and Parasitological Examination

After cleaning the finger surface using sterile cotton wool, a finger prick blood sample was collected. In a single slide labeled with identification number, both thick and thin smears were prepared and stained with 10% Giemsa and observed under the oil immersion microscope objective [10]. The level of parasitemia was expressed as percentage of erythrocytes infected with malarial parasites. Percent parasitemia was calculated by dividing the number of infected RBC by the total number of RBCs indexed and multiplied by 100 [11]. For levels of malarial parasitemia, parasite density was grouped as high parasitemia (>10%), moderate parasitemia (1–10%), and low parasitemia (<1%).

### 3.2. Determination of Hemoglobin Level and Anemia

Finger prick blood samples were collected after rubbing the fingertip using sterile cotton wool and filled the microcuvette. The loaded microcuvette was then inserted into the holder of a portable HemoCue Hb 301 and recorded.

### 3.3. Structured Questionnaires

Sociodemographic data and associated risk factors were collected by trained laboratory technicians using pretested structured questionnaires.

### 3.4. Data Analysis

Data was collected and checked for completeness from each patient and entered to SPSS version 20. The prevalence of malaria was determined as the proportion of those study participants who had positive malaria to total number of participants' blood film examined. Associated risk factors were analyzed by calculating odds ratio with 95% confidence interval. *P* value < 0.05 was recorded as statistically significant.

## 4. Results

### 4.1. Sociodemographic Characteristics

Out of 979 febrile patients, 168/979 (17.2%) of them were malaria positive, and of the total screened cases, 99/168 (58.9%) were males and 69/168 (41.1%) were females. The majority 74/168 (44%) were aged between 15 and 30 years. Most of them 74/168 (44%) were illiterate, and farmers were mainly affected. Prevalence in relation to residence showed that people who live in rural areas (144/168 (85.7%)) were more affected than those who live in urban areas (24/168 (14.3%)) (Table 1).

### 4.2. Malaria Distribution among Health Facilities

The numbers of malaria-infected patients were 77, 57, and 34 from Sire Primary Hospital, Sibu Sire health center, and Chingi health center, respectively. Among the health facilities, the majority of malaria cases were recorded in Sire Primary Hospital (Figure 1).

### 4.3. Sociodemographic Characteristics and *Plasmodium* Species Distribution

The predominant species was *Plasmodium falciparum* (132/168 (78.5%)) followed by *Plasmodium vivax* (27/168 (16.1%)) and mixed infection (9/168 (5.4%)). In the present study, males were more affected than females with a significant difference (*P* = 0.041). Also, people who live in rural areas were more susceptible than those who live in urban areas (*P* = 0.040). Furthermore, the predominant age group was 15-30 years (59/168 (35.1%)) and was statistically significant (*P* = 0.011). The majority of the cases (65/168 (38.7%)) were farmers and statistically significant (*P* = 0.035) (Table 2).

### 4.4. Malaria Parasitemia

Mean parasites/*μ*L of malaria were 85.2 *μ*L and 89.5 *μ*L in male and female, respectively. Mean parasites/*μ*L were the highest in the under-5 age group among the other age groups (Table 3).

### 4.5. Impacts of Malaria Cases on Parasitemia

All febrile patients were examined to determine the level of parasites level among malaria-positive patients. There were 40/168 (23.8%), 106/168 (63.1%), and 22/168 (13.1%) patients with low, moderate, and high parasitemia, respectively. On other hand, the age category less than 5 age group which comprises the large number of patients was with high level of parasitemia which accounts for 20/168 (11.9%), and there was a statistically significant difference (*P* ≤ 0.001). Relatively high level parasitemia was recorded in males compared to females (*P* = 0.510) (Table 4).

### 4.6. Hemoglobin Levels and Malaria-Positive Patients

In malaria-posi

tive patients, mean of hemoglobin decrease from the normal mean in each sex and age is indicated in Table 5.

### 4.7. Impacts of Malaria on the Level of Hemoglobin

In the present study, the range of hemoglobin was from 5 g/dL to 11 g/dL. Out of the total malaria-positive patients, 86/168 (51.2%), 11/168 (6.5%), and 2/168 (1.2) had low, moderate, and severe anemia, respectively. Totally, 4.2% of malaria-positive patients were exposed to low hemoglobin (severe anemia). Both male and female had very low anemia although not statistically significant (*P* = 0.243). All age groups of the study participants had low level of anemia with the highest and lowest recorded from 15-30 years (60/168 (35.7%)) and >49 years (13/168 (7.7%)), and it was statistically significant (*P* value = 0.033) (Table 6).

### 4.8. Malaria Prevalence and Associated Risk Factors

To identify factors associated with malaria among malaria-positive patients, regression analysis was done. As shown in Table 7, in bivariate regression analysis, factors significantly associated with malaria prevalence were sex, age, residence, and working while wearing protective cloth near stagnant water. In multivariate regression analysis, risk factors for malaria prevalence were identified using odds ratio with 95% confidence interval. Regarding the sex of the respondents being female, they were 0.352 times (AOR = 0.352, 95% CI 0.024-0.998) less attacked with malaria when compared with malaria-infected males. The age group between 15 and 30 years (AOR = 0.117, 95% CI 0.015-0.942) was mainly at risk compared to other age groups. Malaria-infected patients who were rural residents are nearly four times (AOR = 3.588, 95% CI 0.088-11.839) at risk of being attacked by malaria when compared to urban residents.

Bed net utilization was considered a backbone of malaria prevention in a community with less cost or free of charge distribution. Among malaria-infected patients, those who did use a bed net were 0.172 times (AOR = 0.172, 95% CI 0.049-0.604) less at risk of being attacked with malaria than those who did not use a bed net in the households properly and continuously. In the current study, 0.162 times (AOR = 2.143, 95% CI 0.042-0.624) of malaria-infected patients did not live around stagnant water when compared to their counterparts. From respondents who did not spray IRS chemical in their house, they were five times (AOR = 5.130, 95% CI 1.088-24.176) vulnerable to malaria than those who sprayed IRS chemical in the room of their house. As means of preventing mosquito bite, wearing protective cloth during working around stagnant water and night was inversely associated with malaria attack. Malaria-infected patients who wear protective cloth were 0.227 times (AOR = 0.227, 95% 0.053-0.976) less to develop malaria when compared to their counterpart who did not wear protective cloth (Table 7).

## 5. Discussion

The study revealed that overall malaria positivity among febrile patients is much less compared to the study conducted in Ethiopia at the Kalala health center where prevalence of malaria cases among febrile patients was 49.4%. In this study, the prevalence of malaria was 17.2%. This finding is much related to the result of a study done in Maputo, Mozambique, among febrile cases where 16% of the patients were malaria positive [14]. In the present study, *P. falciparum* was the dominant malaria species followed by *P. vivax*. This finding is consistent with findings of studies in the high land fringes of Butajira, Jimma, and Harar in Ethiopia where proportions of 62.5%, 76%, and 67.3% were, respectively, reported [15, 16]. Similarly, another study conducted in northern Ethiopia reported 75% of *P. falciparum* and 25% of *P. vivax* cases [17–19]. The variation in the finding could be attributed to the study area, socioeconomic status, and awareness on malaria prevention. Males were more affected than females which could be ascribed to their occupational engagement with agricultural activities during the night when mosquito becomes active and in agreement with earlier studies carried out by Gemechu et al. in Western Ethiopia [7] and Getachew et al. in Northwest Ethiopia [20]. Results of the current study also emphasize that incidence of malaria was higher in rural areas than in urban areas which is in agreement with the study conducted by Dufera et al. in Western Ethiopia [12] and Gomez et al. and Abebe et al. in South West Ethiopia [21, 22].

The present study showed that patients' aged 15-30 years were more vulnerable to malaria which could be ascribed to the fact that people in this age group are in productive age and movable for agricultural activities. This is consistent with the study conducted by Abebe et al. in Northwest Ethiopia [23].

In this study, RBC counts and Hb levels were significantly reduced in high parasitemia patients, which is consistent with previous studies [24] showing a significant increase in the prevalence of anemia with the increase in parasite density. Malaria parasite mean density was higher in febrile patients in the under-5 age group as compared with other age groups and is in agreement with the previous studies conducted in Southern Ethiopia [25] and findings of a meta-analysis [26] which could be related to the premature immunity. The parasite density observed among the study subjects showed that most of the malaria cases were with low level of parasitemia. This suggests that most of the study subjects had a low immune status or had other underlying conditions that predispose them to clinical malaria even at a low parasite density [27]. In general, in the present study, there was low parasite density among febrile adult patients which is in agreement with [28, 29]. In contrast to this study, low level of parasitemia was recorded in children [30, 31]; however, the high parasite densities recorded during the rainy seasons were similar to findings from South East Nigeria [32]. Previous studies have shown that there is a correlation between parasite density and severity of malarial infections [33, 34], and in nonfalciparum malaria, parasitemia rarely exceeds 2%, whereas it can be considerably higher (>50%) in falciparum malaria [35].

The mean Hb level of females was lower than that of males (10.2 g/dL versus 10.9 g/dL) and goes in line with the study conducted by Maina et al. in Western Kenya [36]. Regarding the association between the level of Hb and risks of malaria cases, the level of Hb range was from ≤11 g/dL to ≤5 g/dL. This result is in agreement with the study conducted by Samdi et al. in North Eastern Nigeria [37]. Studies have shown that malaria was estimated to significantly reduce hemoglobin levels, with an overall effect of −7.5 g/dL (95% CI−8.5, −6.5). Acute malaria resulted in a −7.7 g/dL (95% CI −8.8, −6.6) decrease in hemoglobin levels [38].

In the present study, residence and wearing protective clothes while working near stagnant water were significantly associated with malaria prevalence which is similar to the study conducted by Nacher et al. in Southern Ethiopia [39]. A rural resident was at higher risk when compared with those living in urban areas. This finding goes in line with the study conducted by Dondorp et al. and FMoH in Ethiopia [40, 41]. In the present study, habits of not using a bed net had also shown statistically significant association with malaria positivity which is similar to studies conducted by Molla and Ayele in Southern Ethiopia and Delil et al. in the Hadiya Zone, Ethiopia [42, 43].

## 6. Conclusion

The finding of the study indicated that malaria cases among febrile patients visiting Sibu Sire health facilities were 17.2%. In this study, *Plasmodium falciparum* was the most public health problem with higher occurrence in both male and female especially among the 15-30 age category. The burdens of *Plasmodium falciparum* are mostly associated with the occurrence or increase in the load of parasitemia level which leads to the cases for low level of hemoglobin and increase in anemia. The high level of parasitemia and low level of hemoglobin warrant the urgent need of intervention so as to avoid its consequences in increasing anemia especially among the risk groups.

## Figures and Tables

**Figure 1:** Malaria distribution among health facilities

**Table 1:** Sociodemographic characteristics of malaria-positive individuals (*n* = 168).

Characteristics	Response	Number (*n*)	Percentage (%)
Sex	Male	99	58.9
	Female	69	41.1

Age	Under 5	20	11.9
	5-14	30	17.9
	15-30	74	44
	31-49	29	17.3
	>49	15	8.9

Educational status	Illiterate	74	44
	Primary school	56	33.3
	Secondary school	23	13.7
	College and above	15	9

Occupation	Farmer	87	51.8
	Merchant	15	8.9
	Student	29	17.3
	Government employee	4	2.4
	Others^∗^	13	7.7
	No occupation	20	11.9

Residence	Rural	144	85.7
	Urban	24	14.3

^∗^Others = daily labor work, housewife, and private employee.

**Table 2:** Sociodemographic characteristics of the respondents with *Plasmodium* species distribution (*n* = 168).

Demography		*P. falciparumn* (%)	*P. vivaxn* (%)	Mixed *n* (%)	Total *n* (%)	*P* value
Sex	Male	76 (45.2)	17 (10.1)	6 (3.6)	99 (58.9)	0.041
	Female	56 (33.3)	10 (5.95)	3 (1.8)	69 (41.1)	

Age^∗^	Under 5	18 (10.7)	2 (1.2)	0	20 (11.9)	0.011
	5-14	25 (14.9)	5 (3)	0	30 (17.9)	
	15-30	59 (35.1)	13 (7.7)	2 (1.2)	74 (44)	
	31-49	21 (12.5)	6 (3.6)	2 (1.2)	29 (17.3)	
	>49	9 (5.3)	1 (0.6)	5 (3)	15 (8.9)	

Educational status	Illiterate	57 (34)	13 (7.6)	4 (2.4)	74 (44)	0.034
	Primary school	43 (25.6)	9 (5.3)	4 (2.4)	56 (33.3)	
	Secondary school	22 (13.1)	1 (0.6)	0	23 (13.7)	
	College and above	10 (5.6)	4 (2.4)	1 (0.6)	15 (9)	

Occupation	Farmer	65 (38.7)	15 (8.9)	7 (4.2)	87 (51.8)	0.035
	Merchant	12 (7.1)	1 (0.6)	2 (1.2)	15 (8.9)	
	Student	24 (14.3)	5 (3)	0	29 (17.3)	
	Gov. employee	1 (0.6)	3 (1.8)	0	4 (2.4)	
	Others^∗∗^	12 (7.1)	1 (0.6)	0	13 (7.7)	
	No occupation	18 (10.7)	2 (1.2)	0	20 (11.9)	

Residence	Rural	116 (69)	19 (11.3)	9 (5.4)	144 (85.7)	0.040
	Urban	16 (9.5)	8 (4.8)	0	24 (14.3)	

^∗^Age grouping: source [12]; ^∗∗^others = daily labor work, housewife, and private employee.

**Table 3:** Prevalence of mean parasite density of malaria (*n* = 168) malaria-infected patients in Sibu Sire District health care centers.

Variables		Parasite density		Mean parasites/*μ*L
		Minimum	Maximum	
Sex	Male	15	200	85.2
	Female	15	150	89.5

Age	Under 5	75	200	90.9
	5-14	35	150	85.6
	15-30	10	115	45.1
	31-49	35	145	89.3
	>49	40	155	90.7

**Table 4:** Impacts of malaria cases on parasitemia level among malaria-infected patients in Sibu Sire District, 2020 (*n* = 168).

Variables		Parasitemia level			*P* value
		<1% *n* (%)	1-10% *n* (%)	>10% *n* (%)	
Sex	Male	21 (12.5)	66 (39.3)	12 (7.1)	0.510
	Female	19 (11.3)	40 (23.8)	10 (6)	

Age	Under 5	0	0	20 (11.9)	≤0.001
	5-14	5 (3)	25 (14.9)	0	
	15-30	18 (10.7)	55 (32.7)	1 (0.6)	
	31-49	9 (5.3)	20 (11.9)	0	
	>49	8 (4.8)	6 (3.6)	1 (0.6)	

**Table 5:** Mean hemoglobin of malaria-infected patients (*n* = 168) in Sibu Sire District health care centers, 2020.

Variables		Malaria-positive patients		Normal Hgb level in g/dL [13]
		*n* (%)	mean Hgb in g/dL	
Sex	Male	99	10.9	14-18
	Female	69	10.2	12-16

Age	Under 5	20	11	12.5 for both male and female
	5-14	30	11.2	13.5 for both male and female
	15-30	74	10.7	14 for female and 14.5 for male
	31-49	29	10.9	14 for female and 15.5 for male
	>49	15	10.8	14 for female and 15.5 for male

**Table 6:** Impacts of malaria on hemoglobin level among malaria-infected patients in Sibu Sire District, 2020 (*n* = 168).

Variables		Hemoglobin level			*P* value
		>8-11 g/dL	>5-8 g/dL	≤5 g/dL	
		*n* (%)	*n* (%)	*n* (%)	
Sex	Male	86 (51.2)	11 (6.5)	2 (1.2)	0.243
	Female	56 (33.3)	8 (4.8)	5 (3)	

Age	Under 5	17 (10.1)	2 (1.2)	1 (0.6)	0.033
	5-14	26 (15.5)	2 (1.2)	2 (1.2)	
	15-30	60 (35.7)	10 (5.9)	4 (2.4)	
	31-49	26 (15.5)	3 (1.8)	0	
	>49	13 (7.7)	2 (1.2)	0	

**Table 7:** Associated risk factors with malaria among malaria-infected patients, 2020 (*n* = 168).

Risk factors		*n* (%)	COR^∗^	AOR^∗∗^	*P* value
Sex	Male	99 (58.9)	1	1	1
	Female	69 (41.1)	2.844 (1.002-8.077)	0.352 (0.024-0.998)	0.050

Age	Under 5	20 (11.9)	0.632 (0.161-1.388)	0.087 (0.010-0.797)	0.031
	5-14	30 (17.9)	0.847 (0.203-2.324)	0.223 (0.014-1.070)	0.048
	15-30	74 (44)	0.709 (0.242-2.365)	0.117 (0.015-0.942)	0.044
	31-49	29 (17.3)	0.879 (0.223-2.254)	0.187 (0.021-1.669)	0.033
	>49	15 (8.9)	1	1	1

Educ. status	Illiterate	74 (44)	0.283 (0.023-3.425)	3.538 (0.292-12.890)	0.321
	Primary school	56 (33.3)	2.438 (0.491-12.105)	0.410 (0.083-2.037)	0.276
	Secondary school	23 (13.7)	1.135 (0.224-5.738)	0.881 (0.174-4.455)	0.878
	College and above	15 (9)	1	1	1

Residence	Rural	144 (85.7)	0.279 (0.084-2.0.919)	3.588 (0.088-11.839)	0.036
	Urban	24(14.3)	1	1	1

Bed net utilization	Yes	45 (26.8)	5.800 (1.657-20.302)	0.172 (0.049-0.604)	0.006
	No	123 (73.2)	1	1	1

Living around stagnant water	Yes	108 (64.3)	1	1	1
	No	60 (35.7)	6.176 (1.603-23.796)	0.162 (0.042-0.624)	0.008

Application of IRS	Yes	34 (20.2)	1	1	1
	No	134 (79.8)	0.195 (0.041-0.919)	5.130 (1.088-24.176)	0.039

Wearing of protective cloth during night	Yes	10 (6)	4.408 (1.024-18.973)	0.227 (0.053-0.976)	0.046
	No	158 (94)	1	1	1

^∗^Crude odd ratio; ^∗∗^adjusted odd ratio.

## Data Availability

Data can be obtained from the corresponding author upon reasonable request.

## Abbreviations

ACTs: Artemisinin-based combination therapies selective
EMIS: Ethiopian National Malaria Indicator Survey
EPHI: Ethiopian Public Health Institute
FMOH: Federal Ministry of Health
Hb: Hemoglobin
IRS: Indoor residual spraying
ITNs: Insecticide-treated mosquito nets
NSP: National strategic plan
PHEM: Public Health Emergency Management
RLEPOSSD: Rural Land Environmental Protection of Sibu Sire District
SOP: Standard operating procedure.
